# Protease-Activated Receptor 1 Contributes to Microcirculation Failure and Tubular Damage in Renal Ischemia-Reperfusion Injury in Mice

**DOI:** 10.1155/2021/6665714

**Published:** 2021-02-23

**Authors:** Yu Guan, Daisuke Nakano, Lei Li, Haofeng Zheng, Akira Nishiyama, Ye Tian, Lei Zhang

**Affiliations:** ^1^Department of Urology, Beijing Friendship Hospital, Capital Medical University, Beijing, China; ^2^Department of Pharmacology, Kagawa University, Kagawa, Japan; ^3^Division of Kidney Transplantation, Department of Surgery, The Third Affiliated Hospital of Sun Yat-sen University, Guangzhou, China

## Abstract

Ischemia-reperfusion- (IR-) induced kidney injury is difficult to avoid during renal transplantation and robot-assisted partial nephrectomy. Renal IR injury is characterized by tubular damage, microcirculation failure, and inflammation, which coordinately augment renal injury; however, no specific treatment is available for these conditions. Protease-activated receptor-1 (PAR-1) and its ligand, thrombin, are involved in coagulation and were shown to be associated with epithelial cell injury. Here, we hypothesized that PAR-1 exaggerated renal IR-induced tubular cell damage and microcirculation failure and that pharmacological inhibition of PAR-1 by Q94 could prevent these injuries. Renal warm IR increased the expression of PAR-1 in the renal tubules. Q94 attenuated renal IR-induced changes and histopathological damage. Microcirculation failure analyzed by congestion in the histopathology and blood cell flow examined by intravital multiphoton microscopy were suppressed by Q94 treatment. Q94 also dramatically increased tubular cell proliferation despite the lower renal damage. Thrombin suppressed cell proliferation and induced apoptosis in the tubules; these effects were prevented by Q94 treatment. Taken together, PAR-1 was associated with renal IR injury. Inhibition of PAR-1 ameliorated injury possibly by improving renal microcirculation and tubular cell survival/proliferation.

## 1. Introduction

The kidney cannot avoid ischemia-reperfusion (IR) injury during partial nephrectomy and kidney transplantation [1], which is known to result in the retention of metabolic waste products and lead to acute kidney injury (AKI) and AKI-chronic kidney disease (AKI-CKD) [2]. To date, no specific drug therapy is clinically available for AKI and AKI-CKD [3]. Several common pathological changes occur in AKI, such as microcirculation failure [4], including congestion and hemorrhage, and acute tubular necrosis [5]. Therefore, studies have focused on targeting these pathological changes as potential therapeutic candidates. We previously demonstrated that maintaining the peritubular capillaries after renal IR injury reduced capillary congestion and ameliorated the AKI to CKD transition [6]. Acute tubular necrosis may be difficult to treat; thus, regeneration of tubules through tubular cell proliferation may be an important approach for preventing the further loss of renal function [7].

Protease-activated receptor-1 (PAR-1) belongs to the protease-activated receptor (PAR) family and is known to be stimulated by thrombin to induce platelet coagulation. We recently showed that PAR-1 contributed to the development of acutely induced glomerular injury [8]. In addition, thrombin/PAR-1 was reported to play a role in epithelial cell proliferation and apoptosis. Based on these characteristics, we hypothesized that PAR-1 accelerated AKI severity by regulating either peritubular capillary blood coagulation or tubular regeneration. In this study, we examined the role of PAR-1 by using Q-94, a PAR-1-selective negative allosteric modulator, in a mouse renal IR injury model and thrombin-stimulated cultured human tubular cells.

## 2. Materials and Methods

### 2.1. Acute Kidney IR Mouse Model

All animal experiments were performed according to the Institutional Animal Care and Use Committee experimental guidelines of the Capital Medical University. The kidney IR mouse model was established as previously described [8]. Briefly, 8-week-old C57/BL6 male mice were anesthetized by injection of pentobarbital sodium (50 mg/kg; i.p.) and randomly divided into the following groups: sham, I/R+vehicle, and I/R (vehicle: saline 10 mg/kg i.v.)+Q94 (a PAR-1 antagonist at 10 mg/kg i.v.) groups (*n* = 7–8 in each group). For the renal warm IR injury protocol, the mice underwent uninephrectomy to evaluate damage to the renal function; after one week, the renal pedicle was clamped with damage-free vascular clips for 30 min. After reperfusion for 48 h, the mice were sacrificed; their renal tissue samples were collected and fixed in 4% paraformaldehyde solution to prepare paraffin blocks. Plasma was obtained to measure blood urea nitrogen (BUN) and creatinine.

### 2.2. Materials

Q94 was purchased from Tocris Bioscience (Bristol, UK). Other chemicals were obtained from Sigma-Aldrich (St. Louis, MO, USA) unless otherwise stated.

### 2.3. Assay for Creatinine and BUN

Commercial assay kits (Creatinine Assay Kit ab65340; Abcam, Cambridge, UK) were used to measure creatinine. BUN assay kits were purchased from ABSBio™ (UREA NITROGEN Kit, CNHAOBIO, Beijing, China).

### 2.4. Histology

Before embedding in paraffin, the kidney tissue was fixed with 4% paraformaldehyde. Kidney paraffin blocks were cut into 2 *μ*m sections and mounted on slides overnight at 25°C. After deparaffinization, the sections were stained with hematoxylin and eosin (H&E). Images were obtained using a microscope (BX-51/DP-72; Olympus, Tokyo, Japan). As previously described [9], renal-tubule damage was diagnosed based on several histopathological changes, such as tubular dilation, congestion/hemorrhage, brush border loss, tubular cast formation, and cell lysis with sloughed debris in the tubular lumen. Tubular damage was scored according to the percentage of damaged tubules: 0, no damage; 1, <25%; 2, 25–50%; 3, 51–75%; and 4, >75%. Scoring was performed in a blinded manner.

### 2.5. Immunofluorescence and Immunohistochemistry

Sections were prepared as described for the histology (H&E) assay and then incubated with 0.3% hydrogen peroxide for 30 min to block endogenous peroxidases after deparaffinization with xylene. For antigen retrieval, the sections were incubated with proteinase K (DAKO Cytomation, Glostrup, Denmark) for 10 min. After blocking with 10% goat serum, the sections were incubated with primary antibodies overnight at 4°C (anti-Kim 1 antibody, ab47635, Abcam; anti-Ki67 antibody, ab15580, Abcam; anti-PAR-1 antibody, ab32611, Abcam). Following incubation with the primary antibody, the sections were incubated with the secondary antibody at 25°C for 1 h. DAB substrate (DAKO) was used to visualize the immunohistochemistry (IHC) staining results. Fluorescence signals were detected using an Alexa Fluor 594-labeled secondary antibody. Images were captured using a fluorescence microscope (BX51; Olympus) with an appropriate filter. ImageJ software (NIH, Bethesda, MD, USA) was used to analyze the positive areas.

### 2.6. Real-Time PCR

To evaluate the regulation of mRNA expression under these conditions, mRNA was isolated from kidney tissue. A PCR System (7300 Fast Real-Time; Applied Biosystems, Foster City, CA, USA) and Light Cycler Fast Start DNA Master SYBR Green I kit (Applied Biosystems) were used to detect the levels of 18S and PAR-1 mRNA. Primer sequences were as follows: 18S—5′-GTAACCCGTTGAACCCCATT-3′, 5′-CCATCCAATCGGTAGTAGCG-3′; PAR-1—5′-GTTGATCGTTTCCACGGTCT-3′, 5′-GCTGCCTCTGTACCAGGACT-3′. Relative mRNA levels were determined using the 2^−*ΔΔ*Cq^ method. The *ΔΔ*Cq value was calculated using data from the control group.

### 2.7. Surgical Procedure and In Vivo Multiphoton Imaging Settings

The mice were anesthetized with 2% isoflurane (Mylan, Osaka, Japan). After tracheotomy, the jugular vein was cannulated for fluorescent dye injection and infusion of maintenance fluid, which consisted of 1.0 *μ*L/min of 2% albumin in phosphate-buffered saline. The left kidney of each mouse was exteriorized through a small flank incision and attached to a coverslip. The microscope stage and animals were warmed using a heating pad during all experimental procedures. Intravital multiphoton microscopy was performed using an Olympus FV1000MPE multiphoton confocal fluorescence imaging system powered by a Chameleon Ultra-II MP laser at 860 nm (Coherent, Inc., Santa Clara, CA, USA). The microscope objective was a 25x water immersion lens with a 1.05 numerical aperture. The imaging settings for the microscope (gain and offset for all three channels; blue, green, and red) were fixed throughout the experiment. After a 30 min recovery period, rhodamine B-70 kD dextran was injected intravenously, and 3-D z-stack images were taken at depths of 5–50 *μ*m (2 *μ*m apart) from the kidney surface.

### 2.8. Cell Culture

Human kidney 2 (HK2) cells were obtained from the Cell Bank of Academy Sciences (Shanghai, China) and cultured as previously described [10]. The cells were cultured in Dulbecco's modified Eagle's medium supplemented with 10% fetal bovine serum and 1% penicillin-streptomycin in a humidified atmosphere of 95% air and 5% CO_2_ at 37°C.

### 2.9. WST-1 Assays to Evaluate Cell Proliferation

HK2 cells were seeded into 6-well plates at a density of 1 × 10^4^ cells/well. After stimulating the HK2 cells with thrombin, WST-1 assays were performed according to the manufacturer's protocol (catalog #C0035; Beyotime, Shanghai, China) to determine the proliferative ability of cells. After 2 h of incubation with 100 *μ*L WST-1 reagent in each well, the absorbance of the samples was measured using a microplate reader at a wavelength of 450 nm.

### 2.10. Caspase-3 Assay

Caspase-3 activity was measured using a commercially available caspase-3 activity kit (catalog #C1116; Beyotime, Shanghai, China) [11]. Following incubation with the caspase-3 activity kit reagent, the absorbance of the samples was detected using a microplate reader (SpectraMax M2, Molecular Devices, Sunnyvale, CA, USA) at 405 nm according to the manufacturer's instructions.

### 2.11. Data and Statistical Analysis

One-way analysis of variance was used to compare multiple groups, followed by Tukey's multiple comparison test. To compare two individual groups, we used Student's *t*-test. *p* < 0.05 was considered to indicate statistically significant results.

## 3. Results

### 3.1. PAR-1 Expression in the IR Kidney

We first confirmed the expression of PAR-1 and effects of IR on its expression level in the kidney. We observed a nearly 2-fold increase in the expression level of PAR-1 mRNA compared to that in sham surgery mice at 48 h (Figure 1(a)). We also measured the expression of PAR-1 by immunofluorescence at 48 h after IR. PAR-1 was expressed in the tubular cell brush border membrane. The level of PAR-1 fluorescence was upregulated compared to sham group mice (Figures 1(b) and 1(c)). These data suggest that both the localization of PAR-1 in tubular cells and its expression level were upregulated after IR in the kidney.

### 3.2. Renal Function and Histopathological Alterations

We assessed kidney function by detecting the BUN and creatinine levels in the plasma. I/R induced an increase in the levels of BUN and creatinine compared to in mice subjected to sham surgery. Moreover, the IR-induced increase in the BUN level was significantly decreased in Q94-treated mice (Figure 2(a)). The serum creatinine level was inhibited in Q94-treated mice compared to mice subjected only to IR surgery (Figure 2(b)). These data suggest that administration of Q94 can protect kidney function after IR injury.

We also evaluated renal histopathological changes by performing an H&E staining. Renal IR significantly increased cast formation, tubular dilatation, and brush border loss and congestion/hemorrhage in the vehicle-treated mice compared to sham mice. Q94 treatment markedly suppressed these changes induced by IR (Figures 2(c) and 3(a)). Analysis of the H&E staining results between groups revealed the congestion/hemorrhage score and tubular damage score for each group. The Q94 group mice exhibited a much lower score (Figures 2(e) and 3(c)). We also stained Kim-1 as a kidney injury marker of renal tubular cells by IHC [12]. Kim-1-positive areas were increased in the renal tubular area in mice with IR insult, which were significantly suppressed by Q94 (Figures 2(d) and 2(f)). These data suggest that Q94 can suppress kidney tubular damage induced by IR injury.

### 3.3. Abnormal Blood Cell Flow in In Vivo Imaging

PAR-1 and its ligand thrombin play important roles in congestion; Q94 significantly improved congestion. Therefore, we performed intravital imaging by multiphoton microscopy. This enables observation of the blood cell flow in the peritubular capillary in a real-time manner in live mice (Figure 3(c)). Plasma was visualized by 70 kDa dextran conjugated with rhodamine B (Figure 3(d)). Blood cells which do not generate fluorescence in response to the laser were used to excite rhodamine B and depicted as shadows. As shown in Figure 3(e), renal IR disrupted the regular blood cell flow and induced microcirculation failure. Q94 improved peritubular capillary blood cell flow.

### 3.4. Tubular Cell Proliferation after IR Injury

It has been reported that the proliferative regeneration of tubular cells plays an important role in the restoration of the tubular structure and renal function after IR injury. PAR-1 is known to modify the proliferation of epithelial cells when activated by thrombin. We thus detected the proliferation of renal tubular cells in a Ki-67 IHC assay. At 48 h after IR, the number of proliferating Ki-67-positive tubular cells was increased. Q94 further augmented the increased number of Ki-67-positive tubular cells after IR compared to that in only IR-treated mice (Figures 4(a) and 4(b)). In addition, we checked whether the cell proliferation ability was affected by inhibition of PAR-1 in *in vitro* experiments using HK2 cells incubated with thrombin, a PAR-1 agonist. The proliferative activity of HK2 cells was measured by WST-1 assay. As shown in Figure 4(c), the proliferation of HK2 cells was dramatically suppressed following treatment with thrombin. However, this thrombin-induced inhibition was almost abolished by Q94. These data indicate that PAR-1 negatively regulated the proliferation of renal tubular cells, which was almost abolished by the Q94 PAR-1 antagonist.

### 3.5. Renal Tubular Cell Apoptosis

We further examined the apoptosis of renal cells using caspase-3, which is the most important executioner caspase and is activated by both intrinsic and extrinsic pathways during apoptosis [13]. Using thrombin-incubated cultured HK2 cells, we found that thrombin increased the activity of caspase-3. Moreover, administration of Q94 suppressed the activity of caspase-3 (Figure 4(d)). These data suggest that thrombin-induced apoptosis of HK2 cells was inhibited by the Q94 PAR-1 antagonist.

## 4. Discussion

Kidney IR injury is characterized by congestion/hemorrhage, acute tubular necrosis, inflammation, and deposition of cast formation [5]. Here, we showed that inhibition of PAR-1 ameliorated both blood flow-associated change and tubulointerstitial changes. It is well-known that PAR-1 and its ligand, thrombin, play important roles in platelet coagulation, and interference of this system, such as by thrombomodulin [14, 15], may prevent AKI. We showed that PAR-1 inhibition suppressed congestion and improved blood flow in the peritubular capillaries in mice with renal IR injury, suggesting that the PAR-1 system deteriorated microcirculation. In addition, the expression level of PAR-1 was upregulated in the tubules after renal IR injury, indicating that the PAR-1-dependent system in the tubules also exaggerates renal IR injury. It is well established that regeneration of tubular cells is an important process in rebuilding the tubular structure and in recovering renal function after IR injury [16, 17]. Depending on the degree of injury, this repair capacity is not unlimited [18]. Therefore, treatment options to attenuate damage in tubular cells or accelerate their proliferation are urgently needed. Our *in vitro* study showed that PAR-1/thrombin negatively regulated the proliferation of tubular cells, which was in turn accelerated following inhibition of PAR-1. Furthermore, IR injury in mice was shown to increase tubular proliferation at 48 h, with a further increase after PAR-1 inhibition. We found that PAR-1 was increased in the brush border membrane of proximal tubules. As it has been reported that the function of the glomerular filtration barrier is decreased during renal IR injury [19], the filtered thrombin from glomeruli may activate the increased PAR-1, thereby disrupting tubular regeneration.

Our results suggest that the PAR-1/thrombin system suppressed the proliferation of tubular cells and increased apoptosis. However, another study showed opposing effects of PAR-1 when activated by protein C [20, 21]. This apparent conflicting role of PAR-1 may depend on the method of its activation. In our study, a possible explanation for its attributed role was that PAR-1 was activated by filtered thrombin. The size of protein C is over 60 kDa, which is similar to that of albumin [22, 23] and much bigger than that of thrombin (36 kDa). Furthermore, its plasma concentration (<100 nM) is less than 10% of thrombin (>1 *μ*M), indicating that protein C undergoes less filtration and produced a weaker signal compared to thrombin.

Thrombotic episodes are a risk factor for patients in end-stage renal failure [24]. A study showed that PAR-1 deficiency protected against diabetic CKD [25]. In our study, we observed the effect of inhibition of PAR-1 on kidney function at an early phase after IR. In further studies, we intend to develop a chronic kidney IR-induced disease model [2] to evaluate the potential link between PAR-1 with CKD.

In conclusion, we demonstrated that PAR-1 exacerbated microcirculation failure and negatively regulated the proliferation of tubular cells. In contrast, inhibition of PAR-1 contributed to improving microcirculation and the proliferation of tubular cells and after IR, serving as a prominent mechanism of kidney recovery, and should be considered a new strategy in the treatment of AKI.

## Figures and Tables

**Figure 1:** Expression of PAR-1 was upregulated in the kidney. The expression of PAR-1 mRNA was increased in the renal tissues after IR (a). Quantitative analysis of the intensity of anti-PAR-1 fluorescence in sham and IR kidneys (b) and corresponding representative images (c) (*n* = 7-8). Bars = 25 *μ*m. ^∗∗∗^*p* < 0.001 vs. sham. ^∗^*p* < 0.05 vs. sham.

**Figure 2:** Renal function and histopathological changes following inhibition of PAR-1. IR-induced renal dysfunction was significantly suppressed by Q94. Treatment with Q94 inhibited the increase in blood urea nitrogen (BUN) and plasma creatinine (a, b) levels in IR mice (*n* = 7). ^∗^*p* < 0.05 vs. IR+vehicle. H&E staining showed that 30 min of I/R followed by 24 h reperfusion induced much milder tubular damage in IR+Q94 group mouse kidney compared to that in IR+vehicle (c). Analysis of tubular damage score based on H&E images (e) (*n* = 7). ^∗^*p* < 0.05 vs. IR+vehicle. Treatment with Q94 suppressed the increase in the Kim-1-positive area in the kidney of IR-injured mice (d, f) (*n* = 6–7). Bars = 25 *μ*m. ^∗∗^*p* < 0.01 vs. IR+vehicle.

**Figure 3:** Congestion and hemorrhage and microcirculation failure changes following inhibition of PAR-1. IR-induced congestion and hemorrhage were much milder in Q94-treated mouse kidneys. Representative images (a) and corresponding congestion/hemorrhage scores of the renal outer medulla (b). Arrows indicate congestion and hemorrhage. Bars = 50 *μ*m. ^∗^*p* < 0.05 vs. IR+vehicle. (c) Mice were anesthetized, and superficial area of the kidney after 48 h of IR injury was observed. (d) Intravenously injected 70 kDa dextran conjugated with rhodamine B is depicted in magenta. Blood cells are depicted as shadows. Because of the fast blood flow compared to the microscopy time resolution, the shape of blood cell-derived shadows is a thin line. The disrupted capillary blood flow and reduced cell flow make the blood cell shape clearer, and the blood cell-free area is depicted as saturated magenta. (e) Compared to the blood cell flow in the sham group, IR induced abnormal blood cell flow in the peritubular capillaries. In the Q94 group, the blood cell flow was remarkably improved, although there were still some abnormalities, such as reduced plasma flow that made the capillaries thinner. Proximal tubules generate autofluorescence detected in the green channel. Note that current multiphoton microscopy can visualize less than 100 *μ*m depth from the kidney surface; the morphological changes in the tubules typically evident in the outer medullary region are not observable by multiphoton microscopy.

**Figure 4:** PAR-1 inhibition on the proliferation of tubular cells. The proliferation ability of tubular cells was evaluated by Ki-67 IHC staining *in vivo* and *in vitro*. Treatment with Q94 increased the number of Ki-67-positive cells compared to that in I/R + vehicle mouse kidneys (a, b). ^∗∗∗^*p* < 0.001, vs. IR+vehicle. Bars = 50 *μ*m. The proliferation ability of tubular cells *in vitro* was evaluated by WST-1 assay, which showed that Q94 abolished the inhibition of HK2 cell proliferation incubated with thrombin at 72 h (c) (*n* = 7). ^∗∗^*p* < 0.01, vs. thrombin+vehicle. NS.: not significant. Increased activity of caspase-3 was attenuated by Q94 (*n* = 5) (d). Bars = 50 *μ*m. ^∗^*p* < 0.05, vs. thrombin+vehicle.

## Data Availability

The authors confirm that the data supporting the findings of this study are available within the article.
